# *In vivo* and *in vitro* effects of microRNA-27a on proliferation, migration and invasion of breast cancer cells through targeting of SFRP1 gene via Wnt/β-catenin signaling pathway

This article has been retracted.

**DOI:** 10.18632/oncotarget.14662

**Published:** 2017-01-14

**Authors:** Ling-Yu Kong, Mei Xue, Qing-Cai Zhang, Chuan-Fu Su

**Affiliations:** ^1^ Department of Breast, Linyi Cancer Hospital, Linyi 276000, P.R. China; ^2^ Department of Pathology, Linyi Cancer Hospital, Linyi 276000, P.R. China; ^3^ Operating Theatre, Daqing Oilfield General Hospital, Daqing 163000, P.R. China

**Keywords:** microRNA-27a, secreted frizzled-related protein 1, Wnt/β-catenin signaling pathway, breast cancer, proliferation

## Abstract

This study aims to explore the effects of microRNA-27a (miR-27a) targeting of SFRP1 on the proliferation, migration and invasion of breast cancer (BC) cells through the regulation of Wnt/β-catenin signaling pathway. BC and normal breast tissues were obtained from 396 female BC patients and 308 female patients with benign breast lesions respectively. Human normal mammary epithelial (MCF-10A) and BC cell lines (BT-20, MCF-7, T-47D and MDA-MB-231) were cultured. After cell transfection, BC cells were assigned to six groups: control, miR-27a mimics, miR-27a inhibitors, negative control (NC), si-*SFRP1* and si-*SFRP1* + miR-27a inhibitors groups. qRT-PCR assay and Western blot were employed to detect the expressions of miR-27a, SFRP1, Wnt, β-catenin and GSK3β. MTT assay, wound-healing test and Transwell assay were used to test cell proliferation, migration and invasion. BC tissues were found to have higher miR-27a expression and lower SFRP1 mRNA and protein expressions than MCF-10A cells and normal breast tissues. Compared with the control and NC groups, the miR-27a mimics and si-SFRP1 groups exhibited down-regulation of SFRP1, up-regulation of Wnt, β-catenin and GSK3β, and promotion of cell proliferation, migration and invasion. The miR-27a inhibitor group showed up-regulation of SFRP1 and inhibition of cell proliferation, migration and invasion in comparison to the miR-27a mimic group. The si-SFRP1 + miR-27a inhibitors group also exhibited up-regulation of SFRP1 and inhibition of cell proliferation, migration and invasion in comparison to the si-SFRP1 group. miR-27a may activate the Wnt/β-catenin signaling pathway by negatively regulating SFRP1 to promote the proliferation, migration and invasion of BC cells.

## INTRODUCTION

Breast cancer (BC), the most common malignant tumor among women worldwide, accounts for almost 1 in 3 female cancer cases diagnosed in USA and is the second leading cause of cancer-related death in women after lung cancer [1]. BC undergoes a complicated series of stages before it develops fully: usual epithelial hyperplasia, atypical ductal hyperplasia (ADH), ductal carcinoma *in situ* (DCIS) and invasive carcinoma [2]. Currently, for a vast majority of BC patients, mastectomy coupled with radiotherapy is widely put into practice for treatment with a relatively effective result [3]. However approximately10% of women diagnosed with BC exhibited a family history, so further studies concerning BC related genetic variants are necessary [4]. Wacholder et al. revealed that multiple genetic variants were associated with this type of cancer [5]. Although a large number of molecules have been reported as indicators in BC, their precise mechanisms remain to be brought to light.

MicroRNAs (miRNAs), considered a novel class of endogenous molecules, are non-protein coding small RNA molecules that can negatively regulate post-transcriptional gene expression by directly cleaving target mRNA or by inhibiting their translation [6]. A recent study has found that aberrant miRNAs expression is correlated to various human cancers such as colon tumors, breast cancer and lung cancer [7]. MicroRNA-27a (miR-27a), located on chromosome 19, has been shown to have an oncogenic function in carcinomas by targeting prohibitin [8]. In addition, the Wnt/β-catenin signaling pathway has also been found to exert an influence on a variety of cell biological processes, and its over-activation contributes to tumorigenesis, proliferation, and migration in several human cancers including breast cancer [9]. Secreted frizzled-related proteins (SFRPs), serving as endogenous Wnt antagonists by binding directly to Wnts, have been demonstrated to either promote or suppress Wnt/β-catenin signaling depending on the cellular context, concentration and the expression pattern of frizzled receptors. Interestingly, secreted frizzled-related proteins 1 (sFRP1) were reported as a novel target of miR-27a contributing to bone metabolism in hFOB cells [10]. Although several researches have been carried out in order to explore the effect of miR-27a or Wnt/β-catenin signaling pathway on BC and the specific mechanisms [11, 12], it still remains unclear whether the role of miR-27 in proliferation and invasion of BC cells bears a relationship to the Wnt/β-catenin signaling pathway via the regulation of SFRP1. Therefore, this study is intended to shed light on the effects of miR-27a targeting SFRP1 on proliferation, migration and invasion of BC cells through regulating Wnt/β-catenin signaling pathway.

## RESULTS

### The expression of miR-27a in BC tissues and its association to clinicopathological features of BC patients

The levels of GAPDH mRNA in BC cancer and normal breast tissues were 16.2 ± 0.31 and 15.83 ± 0.29, respectively. The Ct values of RNU6 in BC cancer and normal breast tissues were 1.27 ± 0.14 and 1.36 ± 0.12, respectively. Results of RT-PCR revealed a remarkably higher expression of miR-27a in BC tissues than in normal breast tissues (*P* = 0.023) (Figure 1). No significant differences in the expression of miR-27a were found between patients older than 55-year-old and patients younger than 55-year-old, or between premenopausal patients and postmenopausal patients (both *P* > 0.05). Expression of miR-27a was significantly higher in patients with distant metastasis than that in patients without distant metastasis (*P* < 0.001). The relative expression of miR-27a n may be closely correlated to clinical stage and LNM as well as to tumor size (all *P* < 0.001) (as shown in Table 1).

**Figure 1:** The expression of miR-27a in normal breast and BC tissues as detected by qRT-PCR Note: normal breast tissues, n = 308; BC tissues, n = 396. miR-27a, microRNA-27a; BC, breast cancer; qRT-PCR, quantitative real-time polymerase chain reaction.

**Table 1:** Association between miR-27a protein expression and clinicopathological features of patients with BC

Clinicopathological feature	Case	miR-27a protein expression	*P*
Age of onset			0.337
≤ 55 years old	217	2.056 ± 0.710	
> 55 years old	179	2.126 ± 0.735	
Menstruation condition			0.450
Premenopausal	211	2.062 ± 0.708	
Postmenopausal	185	2.117 ± 0.737	
Clinical stages			< 0.001
I stage	38	1.381 ± 0.093	
II stage	235	1.817 ± 0.647	
III stage	123	2.823 ± 0.192	
Tumor size			< 0.001
≤ 2 cm	207	1.862 ± 0.246	
> 2 cm	189	1.921 ± 0.240	
Lymph node metastasis			< 0.001
Yes	186	2.808 ± 0.228	
No	210	1.450 ± 0.259	
Distant metastasis			< 0.001
Yes	118	2.857 ± 0.065	
No	278	1.761 ± 0.618	

Note: miR-27a, microRNA-27a; BC, breast cancer.

### The expression of miR-27a in normal mammary epithelial and BC cell lines

Lower expression of miR-27a was found in the normal mammary epithelial cell line (MCF10A) than in BC cell lines (MDA-MB-231, BT-20, MCF-7 and T-47D). Compared with three other BC cell lines (MDA-MB-231, BT-20 and MCF-7) and with MCF10A cell line, the T-47D cell line exhibited a higher expression of miR-27a (all *P* < 0.05). As a result T-47D cell line was selected for further experiment in this study (Figure 2).

**Figure 2:** The expression of miR-27a in normal mammary epithelial and BC cell lines as detected by qRT-PCR Note: miR-27a, microRNA-27a; BC, breast cancer; qRT-PCR, quantitative real-time polymerase chain reaction; *, compared with T-47D cell line, *P* < 0.05 (MCF10A cells vs. T-47D cells, *P* < 0.001; MDA-MB-231 vs. T-47D cells, *P* = 0.007; BT-20 cells vs. T-47D cells, *P* = 0.021; MCF-7 cells vs. T-47D cells, *P* = 0.003).

### The mRNA and protein expressions of SFRP1 in normal breast and BC tissues, normal mammary epithelial and BC cell lines

The mRNA expression of SFRP1 was significantly lower in BC tissues than in normal breast tissues (*P* = 0.018) (Figure 3A). In line with this finding, the protein expression of SFRP1 in BC tissues was lower than in the normal breast tissues (*P* = 0.029) (Figure 3B, 3C). In contrast to the normal mammary epithelial cell line (MCF10A), BC cell lines (MDA-MB-231, BT-20, MCF-7 and T-47D) had lower mRNA and protein expressions of SFRP1, with the lowest being T-47D cell line (all *P* < 0.05) (Figure 3D, 3E, 3F).

**Figure 3:** The SFRP1 mRNA and protein expressions in normal breast and BC tissues, normal mammary epithelial and BC cell lines **A**. comparison of the SFRP1 mRNA expression between normal breast tissues and BC tissues (*P* = 0.018); **B**. the SFRP1 protein expression in normal breast and BC tissues as detected by Western blot analysis; **C**. comparison of SFRP1 protein expression between normal breast and BC tissues (P = 0.029); **D**. comparison of SFRP1 mRNA expression among normal mammary epithelial and BC cell lines (MCF10A cells vs. T-47D cells, *P* < 0.001; MCF-7 cells vs. T-47D cells, *P* = 0.013; BT-20 cells vs. T-47D cells, *P* = 0.038; MDA-MB-231 vs. T-47D cells, *P* = 0.020); **E**. SFRP1 protein expression in normal mammary epithelial and BC cell lines detected by Western blot; **F**. comparison of SFRP1 protein expression among normal mammary epithelial and BC cell lines (MCF10A cells vs. T-47D cells, *P* < 0.001; MCF-7 cells vs. T-47D cells, *P* = 0.017; BT-20 cells vs. T-47D cells, *P* = 0.042; MDA-MB-231 vs. T-47D cells, *P* = 0.023). Note: BC, breast cancer; SFRP1, secreted frizzled-related protein 1; *, compared with T-47D cell line, *P* < 0.05.

### Relationship between miR-27a and *SFRP1*

In order to verify that miR-27a reduces *SFRP1* levels, TargetScan online database was used. Results indicated that *SFRP1* was the downstream target gene of miR-27a. Meanwhile, *SFRP1* wild and *SFRP1* mutant plasmids were designed to express the wild and mutant loci of miR-27a binding to *SFRP1* (Figure 4A). The results of dual-luciferase reporter gene assay displayed that WIT + mimics group (co-transfection with *SFRP1* wild plasmid and miR-27a) showed an approximate 45% decline in its luciferase activity compared with the WIT + NC, MUT + NC and MUT mimics groups (all *P* < 0.05). The results showed no significant difference in luciferase activity between MUT + NC group and MUT mimics group (*P* > 0.05) (Figure 4B). As derived from the luciferase activity, miR-27a decreased the expression of its potential SFRP1 mRNA target compared to miR-NC (negative control). Therefore, *SFRP1* could be a target gene of miR-27a and its mRNA and protein expressions might be reduced by miR-27a.

**Figure 4:** Effect of miR-27a on SFRP1 as evaluated by TargetScan online database and dual-luciferase reporter gene assay **A**. the binding site of miR-27a to *SFRP1*-3′UTR predicted by TargetScan online database; **B**. comparison of luciferase activity among the four groups detected by dual-luciferase reporter gene assay. Notes: miR-27a, microRNA-27a; SFRP1, secreted frizzled-related protein 1; WIT, wild type; MUT, mutant; *, compared with the WIT + mimics group, *P* < 0.05 (WIT + NC vs. WIT + mimics, *P* = 0.033; MUT + NC vs. WIT + mimics, *P* = 0.036; MUT + mimics vs. WIT + mimics, *P* = 0.028).

### Effect of miR-27a on SFRP1 mRNA and protein expressions in BC cells

The mRNA and protein expressions of miR-27a and SFRP1 in normal breast and BC tissues, normal mammary epithelial and BC cell lines have been shown in the previous results. These indicated an association between the expression level of SFRP1 with miR-27a. T-47D cells were transfected with miR-27a mimics, miR-27a NC, miR-27a inhibitors and si-*SFRP1* respectively, in a further effort to explore the effect of miR-27a on SFRP1 mRNA and protein expressions in BC cells (ensuring first that transfection was successful). The results revealed that compared with control and NC groups, miR-27a mimics and si-*SFRP1* groups showed reduced expressions of SFRP1 mRNA and protein (all *P* < 0.05). The mRNA and protein expressions of SFRP1 in the miR-27a inhibitors group were significantly increased in comparison to these in the miR-27a mimics group (*P* < 0.05). In addition, the mRNA and protein expressions of SFRP1 were obviously increased in the si-*SFRP1* + miR-27a inhibitor group than in the si-*SFRP1* group (*P* < 0.05). No difference in the mRNA and protein expressions of SFRP1 between the control and NC groups (both *P* > 0.05) (Figure 5A, 5B). Thus, these results showed a negative correlation between SFRP1 and miR-27a (Figure 5B).

**Figure 5:** Effect of miR-27a on the SFRP1 mRNA and protein expressions among the six groups **A**. comparison of SFRP1 mRNA expression among six groups; **B**. comparison of SFRP1 protein expression among the six groups; **C**. SFRP1 protein expression among six groups detected by Western blot. Note: miR-27a, microRNA-27a; SFRP1, secreted frizzled-related protein 1; *, compared with the control group, *P* < 0.05 (the miR-27a mimics group vs. the control group, *P* = 0.029 for SFRP1 mRNA, *P* = 0.036 for SFRP1 protein; the miR-27a inhibitors group vs. the control group, *P* = 0.044 for SFRP1 mRNA, *P* = 0.031 for SFRP1 protein; the si-SFRP1 group vs. the control group, *P* = 0.021 for SFRP1 mRNA, *P* = 0.022 for SFRP1 protein); #, compared with the si-SFRP1 group, *P* < 0.05 (the miR-27a inhibitors + si-SFRP1 group vs. the si-SFRP1 group, *P* = 0.023 for SFRP1 mRNA, *P* < 0.001 for SFRP1 protein).

### Effect of miR-27a on the proliferation of BC cells

The miR-27a mimics and si-*SFRP1* groups had increased cell proliferation than the control and NC groups (both *P* < 0.05). When compared with the miR-27a mimics group, the miR-27a inhibitors group showed a more remarkable decrease of cell proliferation (*P* < 0.05). In comparison to the si-*SFRP1* group, the si-*SFRP1* + miR-27a inhibitors group also showed a significantly decreased cell proliferation (*P* < 0.05). No remarkable difference of cell proliferation was observed between the control group and the NC group (Figure 6).

**Figure 6:** Effect of miR-27a on the proliferation of BC cells among the six groups Note: miR-27a, microRNA-27a; BC, breast cancer; *, compared with the control group, *P* < 0.05 (the miR-27a mimics group vs. the control group, *P* = 0.032; the miR-27a inhibitors group vs. the control group, *P* = 0.041; the si-SFRP1 group vs. the control group, *P* = 0.046); #, compared with the si-SFRP1 group, *P* < 0.05 (the miR-27a inhibitors + si-SFRP1 group vs. the si-SFRP1 group, *P* = 0.045).

### Effect of miR-27a on migration and invasion of BC cells

Migration and invasion of BC cells was assessed using wound-healing test (Figure 7A) and Transwell assay (Figure 7C). The results showed that compared with the control and NC groups, the miR-27a mimics and si-*SFRP1* groups exhibited conspicuously increased cell migration and invasion (both *P* < 0.05). In contrast to the miR-27a mimics group, the cell migration and invasion were significantly decreased in the miR-27a inhibitors group (*P* < 0.05). Meanwhile, the migration and invasion of BC cells in the si-*SFRP1* + miR-27a inhibitors group were lower than those in the si-*SFRP1* group (Figure 7B, 7D).

**Figure 7:** Effect of miR-27a on the migration and invasion of BC cells among the six groups **A**. effect of miR-27a on the migration of BC cells among the six groups; **B**. comparison of wound healing rate among the six groups; **C**. effect of miR-27a on the invasion of BC cells among the six groups; **D**. comparison of invasion cell number of BC into Transwell among the six groups. Note: miR-27a, microRNA-27a; BC, breast cancer; *, compared with the control group, *P* < 0.05 (the miR-27a mimics group vs. the control group, *P* = 0.041 for wound-healing rate, *P* = 0.029 for invasive cell number; the miR-27a inhibitors group vs. the control group, *P* = 0.034 for wound-healing rate, *P* = 0.028 for invasive cell number; the si-SFRP1 group vs. the control group, *P* = 0.046 for wound-healing rate, *P* = 0.035 for invasive cell number); #, compared with the si-*SFRP1* group, *P* < 0.05 (the miR-27a inhibitors + si-SFRP1 group vs. the si-SFRP1 group, *P* = 0.021 for wound-healing rate, *P* = 0.038 for SFRP1 invasive cell number).

### Effect of miR-27a on Wnt/β-catenin signaling pathway through targeting SFRP1

It has been reported that SFRP1 is an antagonist of Wnt/β-catenin signaling pathway [13], and the mRNA and protein expressions of SFRP1 were regulated by miR-27a. The expressions of Wnt, GSK3β and β-catenin in BC tissues were abnormally over-expressed. To explore regulatory effect of miR-27a on Wnt/β-catenin signaling pathway, the mRNA and protein expressions of β-catenin, GSK3β and Wnt were detected using qRT-PCR and Western blot. The results revealed that both the miR-27a mimics and si-*SFRP1* groups had evidently higher mRNA and protein expressions of β-catenin, GSK3β and Wnt than the control and NC groups. Thus, miR-27a might activate the expressions of β-catenin, GSK3β and Wnt in the Wnt/β-catenin signaling pathway. This was supported by the increased levels of transcription and translation (all *P* < 0.05). Furthermore, the mRNA and protein expressions of β-catenin, GSK3β and Wnt were markedly lower in miR-27a inhibitors group than in the miR-27a mimics group (all *P* < 0.05). Compared with the si-*SFRP1* group, mRNA and protein expressions of β-catenin, GSK3β and Wnt in the signaling pathway were remarkably up-regulated in the si-*SFRP1* + miR-27a inhibitors group (Figure 8A, 8B, 8C). Due to β-catenin's wide distribution in the cytoplasm and nucleus, the possible effects of miR-27a on the expressions of β-catenin in the cytoplasm and nucleus were also explored. The results demonstrated that the protein expression of β-catenin either in cytoplasm or in nucleus was increased by miR-27a (Figure 8D). These results contributed to the conclusion that miR-27a promoted the expression of β-catenin, GSK3β and Wnt in Wnt/β-catenin signaling pathway via targeting SFRP1.

**Figure 8:** Effect of miR-27a on Wnt/β-catenin signaling pathway through targeting SFRP1 **A**. comparisons of mRNA expressions of β-catenin, GSK3β and Wnt among the six groups (the miR-27a mimics group vs. the control group, *P* = 0.019 for β-catenin mRNA, *P* = 0.026 for GSK3β mRNA, *P* = 0.037 for Wnt mRNA; the miR-27a inhibitors group vs. the control group, *P* = 0.011 for β-catenin mRNA, *P* = 0.017 for GSK3β mRNA, *P* = 0.016 for Wnt mRNA; the si-SFRP1 group vs. the control group, *P* = 0.023 for β-catenin mRNA, *P* = 0.032 for GSK3β mRNA, *P* = 0.042 for Wnt mRNA; the miR-27a inhibitors + si-SFRP1 group vs. the si-SFRP1 group, *P* = 0.039 for β-catenin mRNA, *P* = 0.043 for GSK3β mRNA, *P* = 0.039 for Wnt mRNA); **B**. protein expressions of β-catenin, GSK3β and Wnt among the six groups detected by Western blot; **C**. comparisons of mRNA expressions of β-catenin, GSK3β and Wnt among the six groups (the miR-27a mimics group vs. the control group, *P* = 0.027 for β-catenin protein, *P* = 0.035 for GSK3β protein, *P* = 0.046 for Wnt protein; the miR-27a inhibitors group vs. the control group, *P* = 0.022 for β-catenin protein, *P* = 0.038 for GSK3βprotein, *P* = 0.033 for Wnt protein; the si-SFRP1 group vs. the control group, *P* = 0.031 for β-catenin protein, *P* = 0.039 for GSK3β protein, *P* = 0.040 for Wnt protein; the miR-27a inhibitors + si-SFRP1 group vs. the si-SFRP1 group, *P* = 0.042 for β-catenin protein, *P* = 0.046 for GSK3β protein, *P* = 0.044 for Wnt protein); **D**. protein expression of β-catenin in cytoplasm and nucleus among the six groups detected by Western blot. Notes: miR-27a, microRNA-27a; SFRP1, secreted frizzled-related protein 1; GSK3β, glycogen synthase kinase-3β; *, compared with the control and NC groups, *P* < 0.05; #, compared with the si-S*FRP1* group, *P* < 0.05.

## DISCUSSION

This study aimed to explore the effect of miR-27a on the proliferation, migration and invasion of BC cells, which activated Wnt/β-catenin signaling pathway via targeting SFRP1, so as to provide a theoretical basis for the development of targeted therapy for BC. In our study, we found that the expression of miR-27a in BC tissues was significantly higher than that of normal breast tissues. Compared to MCF10A cell line, miR-27a expression in BC cell lines (BT-20, MCF-7, T-47D and MDA-MB-231) was increased, especially in T-47D cell line. Thus, miR-27a was over-expressed in BC cells and tissues. For our analyses we applied the SYBR Green method to detect miR-27a expression, because this method, when using high performance primers, proper protocols and material, can provide data as precise as the TaqMan method with less cost requirements and simpler operation [14]. Therefore, we applied SYBR Green method to detect the relative expressions of miR-27a. It has been shown in past research that miR-27a was greatly expressed in estrogen receptor (ER)-negative MDA-MB-231 BC cells, and indirectly regulated specific protein expressions in MCF-7 BC cells [15, 16]. Study had also indicated that miR-27a was highly expressed in BC cells through observation, where miR-27a could lead to cell cycle arrest by inhibiting the expression of its downstream genes [11]. Consistent with these studies, our results showed a high expression of miR-27a in BC cells. The expression level of miR-27 was related to LNM, late clinical stage and poor prognosis, indicating that it could be used as a molecular prognostic marker for BC progression [17]. In line with these findings, the expression of miR-27a was closely associated with clinical stage, lymph node metastasis (LNM) and tumor size in this study. Some evidence had showed that miRNA played an important role in the occurrence of tumor, development, proliferation, invasion, metastasis, and so on [18, 19]. The miR-27a promotes proliferation, migration and invasion of human osteosarcoma cells, perhaps through the targeting of mitogen activated protein kinase kinase 4 (MAP2K4) [20]. However, limited studies concerned the effects of miR-27a on proliferation of BC cells, and none mentioned the specific mechanism. This study found that miR-27a promoted proliferation, migration and invasion of BC cells. Compared with the control and NC groups, the miR-27a mimics exhibited significantly accelerated proliferation, migration and invasion of BC cells. In order to explore the potential mechanism by which miR-27a affects these of BC cells through targeting SFRP1, the miR-27a inhibitors and si-SFRP1 were selected for cell transfection.

The present study illustrated that the expression of SFRP1 mRNA and protein in BC cells and tissues was significantly lower than these of normal breast tissues and MCF10A cells. A study concerning glioma showed that SFRP1 was a direct target of miR-27a, and proved that expression levels of SFRP1 were inversely associated with those of miR-27a [21]. This study found *SFRP1* could be a target gene of miR-27a and its mRNA and protein expressions might be negatively regulated by miR-27a. Additionally, miR-27a may promote the differentiation of osteoblasts through reducing the expression of SFRP1 at the transcriptional level [10]. The results indicated that inhibiting SFRP1 could increase the proliferation, migration and invasion of BC cells. Previous studies have shown that the proliferation, migration and invasion of gastric cancer cells were inhibited after miR-27a was silenced or down-regulated [22]. Similarly in the present results, the inhibition of miR-27a contributed to increased SFRP1 mRNA and protein expressions. As an antineoplastic factor, miRNA-27a inhibited the Wnt/β-catenin signaling pathway to influence proliferation, migration and invasion ability of glioma cells [21]. The β-catenin signaling pathway was an important part of the Wnt signaling pathway, which influenced the expression of the downstream gene [23]. This proved that Wnt signaling played a fundamental role in the development and maintenance of many organs [24]. During both proliferation and osteogenic differentiation, miR-27a could significantly decrease SFRP1 expression by activating Wnt/β-catenin signaling, which leading to an accumulation of β-catenin [10]. The present study revealed that miR-27a increased expressions of related proteins to Wnt/β-catenin signaling pathway, such as β-catenin, GSK3β and Wnt. The inhibition of SFRP1 also caused increased mRNA and protein expressions of β-catenin, GSK3β and Wnt. After inhibiting miR-27a, these expressions were suppressed. Therefore, the role of miR-27a might be achieved through targeting SFRP1, which further activated the Wnt/β-catenin signaling pathway.

In conclusion, this study found that miR-27a was highly expressed in BC, which activated Wnt/β-catenin signaling pathway through negatively regulating SFRP1 to promote the proliferation, migration and invasion of BC cells. However, further evidence of this mechanism should be sought in the future study with larger samples. Therefore more studies are necessary to be conducted to provide a theoretical basis of miR-27a as a novel target for the diagnosis and treatment of BC.

## MATERIALS AND METHODS

### Ethics statement

The study was approved by clinical experiment ethical committee of Linyi Cancer Hospital, and all participants were informed and gave written consent.

### Subjects

A total of 396 female breast cancer (BC) patients were selected from those who underwent surgery (modified radical mastectomy or radical mastectomy for breast cancer) at the Oncology department of Linyi Cancer Hospital from Oct, 2013 to Nov, 2015. Inclusion criteria: Inclusion criteria: all patients were diagnosed with BC by preoperative mammography, color ultrasonography and fine-needle aspiration cytological examination, and confirmed by intraoperative frozen-section examination and postoperative pathological analysis; patients did not receive anti-cancer treatment of chemotherapy or radiotherapy before operation; patients did not have other systemic diseases, such as gastrointestinal cancer, liver cancer, nasopharyngeal carcinoma, lung cancer, endometrial cancer, cervical cancer, leukemia, chronic gastroenteritis and so on, which were primarily identified in accordance with medical history, routine blood, urine and stool examinations, liver and renal function tests, observation of bleeding time and clotting time, ultrasound B-mode examination and menstrual conditions (vaginal secretions) of patients and so on. If any doubt existed, further exclusion was performed with specific examination. Thorough medical history and follow-up information of all patients was requested. Exclusion criteria: patients with incomplete clinical data collection or lack of clinical data; patients had chemotherapy, radiotherapy or other treatment before operation. The ages of these patients ranged from 24 to 86 years old, with an average age of 50.36 ± 19.86 years. There were 211 premenopausal patients and 185 postmenopausal patients. There were 189 patients with tumor size > 2 cm, and 207 patients with tumor size ≤ 2 cm. There were 186 patients with lymph node metastasis (LNM) and 210 patients without LNM. There were 118 patients with distant metastasis and 278 patients without distant metastasis. According to the UICC tumor node metastasis (TNM) staging for BC (2003) [25], there were 38 patients with stage I BC, 235 patients with stage II BC and 123 patients with stage III BC (Table 1). Normal breast tissues obtained from 308 female patients with benign breast lesions were selected as a control.

The fresh BC tissues (2 to 5 g per individual) were collected once the surgery was over. The normal breast tissues (2 to 3 g per individual) were collected at 1 to 2 cm distances from the benign breast lesions. Both BC and normal breast tissues were stored in liquid nitrogen containers, and then cryopreserved in a -80°C freezer.

### Cell culture

Immortalized mammary epithelial cell line (MCF-10A) and BC cell lines (BT-20, MCF-7, T-47D and MDA-MB-231) were all bought from American Type Culture Collection (ATCC). MCF-10A cells were cultured in Dulbecco minimum essential medium (DMEM)/F12 which contained 5% horse serum, 20 ng/ml Epidermal Growth Factor (EGF), 0.1 mg/ml Cholera Toxin (CT), 10 mg/ml insulin and 500 ng/ml hydrocortisone. BC cell lines were all incubated in DMEM which contained 10% inactivated fetal calf serum, 100 units/ml penicillin plus 100 mg/ml streptomycin. DMEM was kept in a 5% CO_2_ incubator at 37°C. Cell digestion with 0.25% trypsin and subculture were conducted after cells covered 80% of the images under microscope. The quantitative real-time polymerase chain reaction (qRT-PCR) was performed to detect miR-27a expression in normal mammary epithelial and BC cell lines.

### Oligonucleotide synthesis and vector construction

MiR-27a mimics, inhibitors and its negative control (NC) oligonucleotides were synthesized by and siRNA *SFRP1* (si-*SFRP1*) was bought from Shanghai GenePharma Co., Ltd (Shanghai, China). The oligonucleotide sequences were shown in Table 2. In order to explore the regulation mechanism of miR-27a on SFRP1 expression, the *SFRP1* 3′-UTR segment, containing miR-27a binding sites in 3′-UTR region, was amplified. Then the amplified segment was implanted into the pGL3 vector to construct pGL3-WT-*SFRP1*-3′- UTR (*SFRP1* wild) plasmid and pGL3-MUT-*SFRP1*-3’-UTR (*SFRP1* mutant), which were the wild and mutant loci of miR-27a binding to *SFRP1*.

**Table 2:** MiRNA oligonucleotide sequences for cell transfection

Oligonucleotide	Sequence
miR-27a mimics	5′-AAGUGUCACCGAUUCAAGGCG-3′
miR-27a inhibitors	5′-GCGGAACUUAGCCACUGUGAA-3′
NC	5′-UUCUCCG AACGUGUCACGUTT-3′

Note: NC, negative control.

### Cell transfection

BC cells were putted on the plate and routinely incubated twenty-four h before cell transfection. One hour before transfection, medium was exchanged with an addition of 2 mL routine DMEM into each well. All medium in the plate was suctioned out and added with the transfection compounds which were prepared using a Lipofectamine 2000 (Invitrogen) kit. Then cells were incubated and cultured at 37°C. After that, BC cells were transfected and assigned to six groups: control group, miR-27a mimics group (transfected with miR-27a mimics), miR-27a inhibitors group (transfected with miR-27a inhibitors), negative control (NC) group (transfected with negative control oligonucleotide), si-*SFRP1* group (transfected with si-*SFRP1*) and si-*SFRP1* + miR-27a inhibitors group (co-transfected with both si-*SFRP1* and miR-27a inhibitors). BC cells in these groups were stored for later experiments such as qRT-PCR, Western blot, MTT assay and Transwell assay. Aside from this, BC cells were transfected with *SFRP1* wild/mutant, miR-27a mimics/NC, and dual firefly and Renilla luciferase plasmid. They were divided into four groups: WIT + mimics group (co-transfected with *SFRP1* wild and miR-27a mimics), WIT + NC group (co-transfected with *SFRP1* wild and negative control oligonucleotide), MUT + mimics group (co-transfected with *SFRP1* mutant and miR-27a mimics), and MUT + NC group (co-transfected with *SFRP1* mutant and negative control oligonucleotide). Luciferase activity was detected with dual-luciferase reporter gene assay (Promega Corporation, Madison, WI, USA). Successful transfection was ensured before cells were used for biological detection.

### Luciferase-reporter gene assay

The target gene of miR-27a was predicted by online software TargetScan 7.1 (http://www.targetscan.org/vert_71/). DNA fragments containing miR-27a-binding site in the 3’-untranslated regions (3’-UTR) of *SFRP1* and fragments containing the mutant miR-27a-binding site were separately inserted into the luciferase reporter gene plasmid to obtain the *SFRP1*-WT (wild type) and *SFRP1*-MUT (mutant type) plasmids. Afterwards, miR-27a mimics and *SFRP1*-WT/*SFRP1*-MUT plasmids were co-transfected into 293T cells, and the luciferase activities in transfected cells were detected using luciferase assay. Additionally, 293T cells were co-transfected with negative control (NC) oligonucleotide and *SFRP1*-WT/*SFRP1*-MUT plasmids as a control.

### qRT-PCR

According to the manufacturer's instructions of miRNeasy Mini kit (Qiagen, Hilden, Germany), miRNAs were extracted from normal breast and BC tissues, mammary epithelial and BC cells, and RNAs in these tissues and cells were also manually extracted with TRIzol (Invitrogen, Inc., Carlsbad, CA, USA). RNA concentrations were detected by NanoDrop2000 (Thermo Fisher Scientific, Massachusetts, USA), after which RNA samples were stored at -80°C. According to gene sequences published in GenBank, primers as follows (Table 3) were designed using Primer5.0 software, and synthesized by Shanghai GenePharma Co., Ltd (Shanghai, China). The miRNA reverse transcription was performed as the instruction of One Step PrimeScript® miRNA cDNA Synthesis Kit (Perfect Real Time) (Takara Biotechnology Ltd., Dalian, China). After the addition of prepared reagents, samples were reacted at 37°C for 1 h (poly (A) tailing reaction and reverse transcription reaction), and heat-shocked at 85°C for 5 s (enzyme inactivation reaction). Reaction condition of miRNA real time PCR: pre-denaturation at 95°C for 10 s, and 40 cycles (annealing at 95°C for 5 s and extension at 60°C for 20 s). The real time PCR for non-miRNA detection was performed as the instructions of One Step SYBR® PrimeScript® PLUS RT- PCR Kit (Takara Biotechnology Ltd., Dalian, China). The reaction condition: pre-denaturation at 42°C for 5 min and denaturation at 95°C for 10 s, and followed by 40 cycles (annealing at 95°C for 5 s and extension at 60°C for 30 s). With *GAPDH/RNU6* as internal controls, the reliability of real-time PCR was evaluated by the solubility curve. The (cycle threshold) Ct value (power amplification knee point) was gotten, and the relative expressions of target genes were calculated by 2^-△△^Ct [26]. All these experiments were repeated three times.

**Table 3:** Primer sequences for quantitative real-time polymerase chain reaction

Gene	Forward primer sequence (5′-3′)	Reverse primer sequence (5′-3′)
miR-27a	TTCACAGTGGCTAAG	CCAGTGCAGGGTCCGAGGT
U6	GCTTCGGCAGCACATATACTAAAAT	CGCTTCACGAATTTGCGTGTCAT
SFRP1	AAAGCAAGGGCCATTTAGATTAG	TTCTGGGCTTGACCTTAATTGTA
β-catenin	AACAGGGTCTGGGACATTAGTC	CGAAAGCCAATCAAACACAAAC
GSK3β	GGACTAAGGTCTTCCGACCC	TAGCATCTGACGCTGCTGTG
Wnt	CTGCAACTGCACCTTCCACT	ATGACACCATCAGGAGCCGA
GAPDH	TCGACAGTCAGCCGCATCTTCTTT	ACCAAATCCGTTGACTCCGACCTT

### Western blotting

Tissues were extracted and their protein concentrations were tested according to bicinchoninic acid (BCA) kit (Wuhan Boster Company, Wuhan, China). After adding loading buffer, the extracted proteins were heated at 95°C for 10 min. A total of 30 ug loading buffer and proteins were added to each well of the loading plate, which were then isolated with 10% polyacrylamide gel electrophoresis (Wuhan Boster Company, Wuhan, China) at 80 v to 120v. Isolated proteins were transferred to membrane using a wet-transferring method at 100 v for 45 to 75 minutes. After this polyvinylidene fluoride (PVDF) transmembrane and 5% bovine serum albumin (BSA) were added, followed by sealing for 1 h at room temperature. Next, the primary antibodies were added to samples: *SFRP1* (ab4193, diluted at 1: 600), *Wnt* (ab15251, diluted at 1: 1000), *GSK3β* (ab32391, diluted at 1: 1000), *β-Catenin* (ab16051, diluted at 1: 1000), *β-tubulin* (ab4074, diluted at 1: 1000, and *β-actin* (ab16039, diluted at 1: 1000), all bought from Abcam Inc., Cambridge, MA, USA. After this samples were stored overnight at 4°C. Having been rinsed with Tris-buffered saline with Tween 20 (TBST) 3 times (5 min per time), corresponding second antibodies (diluted at 1: 2000, Wuhan Boster Company, Wuhan, China) were added into samples, and this was followed by incubation for 1 h at room temperature. After the membrane was washed 3 times (5 min per time), developing was performed with chemiluminescence reagents. With *β-tubulin* and *β-actin* as internal control, the gray-level histogram and protein image were made on the basis of WB results. All of these experiments were repeated three times.

### MTT assay

Transfected BC cells were diluted to a certain concentration and then were placed over a 96-well plate, at a density of 5 × 10^3^ cells per well. Each well was inoculated with 100 μL cell suspension, apart from one blank well (instead with 100 μL medium containing 10% fetal bovine serum). Then they were cultured in a CO_2_ incubator at 37°C. After 24 h, 48 h, 72 h and 96 h of culture, the proliferation of BC cells was detected by MTT assay. With an addition of 20 μL 3-(4,5-Dimethylthiazol-2-yl)-5-(3-Carboxymethoxyphenyl)-2-(4-Sulfophenyl)-2H-Tetrazolium, Inner Salt (MTS) reagent (Promega Corp., Madison, Wisconsin, USA) to each well, cells were then cultured in an incubator for 1 ~ 4 h. After that, the optical density (OD) at 570 nm of each well was obtained with a microplate reader (Biotek Instruments, Inc., Vermont, USA). The target wavelength was 570 nm, and the reference wavelength was 630 nm. The cell proliferation was evaluated by OD value. All of these experiments were repeated three times.

### Wound-healing test

After transfection in 6-well plate, BC cells were incubated at 37°C. When cells fully covered the plate bottom, a line was lightly drawn in each well with a sterilized tip, ensuring the width of each line was same. A mark was left on the cap of the 6-well plate in order to make sure the same visual field in the photograph, and then photos were taken and recorded as 0 h. After a 24 h incubation at 37°C, cell culture fluids were suctioned out and discarded. The 6-well plate was washed 3 times with PBS to remove any cell debris caused by scratching. Then cells were put into serum-free medium for photographing, and recorded as 24 h. Photographs were taken with Olympus Inverted Microscope (Olympus Optical Co., Ltd, Tokyo, Japan) with 6 visual fields at a fixed location. The healing rate was calculated with the ImageTool software (Bechtel Nevada, Los Alamos Operations, USA). Healing rate = (the width of scratch at 0^th^ h - the width of scratch at 24^th^ h)/the width of scratch at 0^th^ h × 100%. All of these experiments were repeated three times.

### Transwell assay

Each Transwell chamber (Corning Glass Works, Corning, New York, USA) was added with matrigel (3.9 mg/ml, 60~80 μl), and incubated at 37°C. When the matrigel was coagulated, chambers were taken out and put into a 24-well plate. After the medium was pre-warmed in the incubator, the pre-warmed mediums (0.5 mL per chamber) were separately added into upper and lower chambers. Then the chambers were put into the incubator for a 2-h hydration, followed by the liquid being suctioned out from upper and lower chambers and being discarded. The cell suspension (5 × 10^4^ cells/ml) was prepared after digestion. A total of 0.5 ml complete medium was extracted and put into a 24-well plate, and then the hydrated chamber was transferred into the 24-well plate, avoiding bubble formation. A total of 0.5 ml cell suspension was extracted and put into the chamber, followed by incubation at 37°C for 24 h. The liquid in upper and lower chambers was suctioned out and discarded. Cotton swabs were used to clean the cells on the surface of the upper chamber of the Transwell membrane. After three PBS washed, the transferred cells were fixed with ice-cold methanol for 30 min. Cells were then dyed with 0.1% crystal violet for 10 min. After this, cells were washed with running water until no extra crystal violet remained, and were air dried. Finally, data were recorded through observation and photography under a microscope. Photographs were captured using Olympus Inverted Microscope (Olympus Optical Co., Ltd., Tokyo, Japan) with 6 visual fields at a fixed location. A hit counter was applied to count the number of cells transferred onto Transwell lower chamber. All of these experiments were repeated three times.

### Statistical analysis

All data were analyzed by SPSS version 18.0 statistical software (SPSS, Chicago, IL, USA). Measurement data were expressed by mean ± standard deviation. The *t* test was used for comparisons between two groups. One-way analysis of variance (One-Way ANOVA) was applied for comparisons between multiple groups. Enumeration data were expressed by percentage or ratio, and detected by chi-square test. Statistical significance was assumed for *P* < 0.05.
